# Ankle-Injury Patients Perform More Microadjustments during Walking: Evidence from Velocity Profiles in Gait Analysis

**DOI:** 10.1155/2022/3057270

**Published:** 2022-01-06

**Authors:** Xin Liu, Bin Zheng, Qinwei Guo, Yuanyuan Yu, Zhongshi Zhang, Aziguli Wulamu, Dezheng Zhang

**Affiliations:** ^1^School of Computer and Communication Engineering, University of Science and Technology Beijing, Beijing, China 100083; ^2^Surgical Simulation Research Laboratory, Department of Surgery, University of Alberta, Edmonton, Alberta, Canada T6G 2E1; ^3^Beijing Key Laboratory of Knowledge Engineering for Materials Science, Beijing, China 100083; ^4^Institute of Sports Medicine, Peking University Third Hospital, Beijing, China 100191; ^5^Department of Biological Sciences, University of Alberta, Edmonton, Alberta, Canada T6G 2E9

## Abstract

**Introduction:**

We evaluated the velocity profiles of patients with lateral collateral ligament (LCL) injuries of the ankle with a goal of understanding the control mechanism involved in walking.

**Methods:**

We tracked motions of patients' legs and feet in 30 gait cycles recorded from patients with LCL injuries of the ankle and compared them to 50 gait cycles taken from normal control subjects. Seventeen markers were placed on the foot following the Heidelberg foot measurement model. Velocity profiles and microadjustments of the knee, ankle, and foot were calculated during different gait phases and compared between the patient and control groups.

**Results:**

Patients had a smaller first rocker percentage and larger second rocker percentage in the gait cycle compared to controls. Patients also displayed shorter stride length and slower strides and performed more microadjustments in the second rocker phase than in other rocker/swing phases. Patients' mean velocities of the knee, ankle, and foot in the second rocker phase were also significantly higher than that in control subjects. *Discussion*. Evidence from velocity profiles suggested that patients with ligament injury necessitated more musculoskeletal microadjustments to maintain body balance, but these may also be due to secondary injury. Precise descriptions of the spatiotemporal gait characteristics are therefore crucial for our understanding of movement control during locomotion.

## 1. Introduction

Many individuals experience ankle twists, which can cause ligament damage around the affected ankle. Lateral collateral ligament (LCL) injuries of the ankle occur in one of every 10,000 people each day worldwide, ranking highest among trauma cases in emergency departments [1, 2]. Symptoms such as pain, swelling, and limited motion are present in 40% of individuals who have experienced LCL injuries. Moreover, recurrences of LCL injuries are high, and approximately 18% of patients will damage their ligament again within a year after the first LCL injury due to difficulty in posture control [3]. Frequent ligament injuries and functional limitations to their lower extremities will then affect a patient's quality of life [4, 5]. In some cases, surgical treatment and long-lasting rehabilitation are required.

To improve our understanding of the mechanisms underlying LCL injuries, gait analysis is necessary. Spatiotemporal characteristics of the foot and ankle allow quantitative assessments of gait and the choice of interventions [6]. These detailed descriptions can also assist physiotherapists to improve their rehabilitation treatment and help designers develop rehabilitation-assistive products [7–9]. Gait analysis using motion tracking data allows scientists to understand posture control and force application of the foot during walking [10, 11]. For example, Chinn et al. found that subjects with ankle instability experienced more inversions during jogging than walking [12]. Moisan et al. reported that subjects with chronic ankle instabilities displayed ankle inversion and laterally deviated the center of pressure during the stance phase during walking and running [13]. However, there are few reports on the velocity profiles of LCL injury patients during gait analysis, and fewer studies have reported acceleration profiles [14].

We believe that examination of the acceleration and velocity profile is important as it describes the strategy of movement speed, which provides critical information, to quantitatively measure stance and swing phases during a gait cycle. Using velocity and acceleration, we revealed underlying pathologic changes caused by ligament injuries around the ankle and foot, in addition to the mechanisms underlying stability control in LCL-injury patients.

In this study, we examined velocity characteristics of patients diagnosed with grade III LCL injuries; data were compared to control (healthy) subjects during the entire gait cycle. Specifically, we tracked patient leg movements in the gait analysis laboratory using the Heidelberg foot measurement model (HFMM) and calculated spatiotemporal features during stance and swing phases. With respect to selected points, such as the knee, ankle, back foot, and front foot, we examined acceleration and velocity profiles.

We used microadjustments, where the acceleration dropped to zero, to describe movement speed changes based on data presented in participants' acceleration profiles. We hypothesized that patients with ligament injury would (a) exhibit a shorter stance phase due to the pain surrounding their ankles, (b) manifest a relatively slower velocity, and (c) display an increasing number of adjustments during walking due to impaired proprioception and neuromuscular control, as compared to control subjects.

## 2. Methods

### 2.1. Participants

This study was conducted at the motion analysis laboratory of the Peking University Third Hospital. The Institutional Research Board of the Peking University Third Hospital reviewed and approved the protocol. Each participant provided informed written consent before entering the study.

We recruited patients who met the following criteria: (1) diagnosed with grade III LCL injuries of the ankle (severe and complete rupture of the ligament fibers) without bone fracture (by X-ray inspection); (2) presented with multiple lateral ankle sprains that required surgical treatment; (3) had a recent sprain that occurred at least three months previously, as we examined the long-term impact of ligament injuries on patient mobility; and (4) age fell in the range of 18 to 40 years.

A patient with these criteria was excluded: (1) a combination of ankle osteoarthritis or cartilage injury; (2) LCL injury was combined with knee/hip osteoarthritis, ligament injuries, or cartilage injuries; (3) had neurologic abnormality; and (4) condition was accompanied by other serious medical diseases that reduced mobility.

According to the inclusion and exclusion criteria above, three patients and three paired healthy adults were recruited. The healthy adults who served as control subjects were enrolled from our hospital's students and staff who did not exhibit known foot or ankle abnormalities, previous injuries, or surgeries.

In this study, we used both left and right limbs from control subjects and the affected side including 2 right limbs and 1 left limb from patients to obtain the acceleration and velocity profile.

### 2.2. Procedure

Before data acquisition, we read the instructions to each subject, ensuring them of familiarity with the task. Subjects were required to walk barefoot along a 10-meter flat path at their own chosen speed (Figure 1(a)), wearing dark sports shorts and T-shirts. A total of 17 reflective markers (13 of 9 mm and 4 of 14 mm in size) were placed on the key bony landmarks of each participant's leg (Figure 1(b)) following the HFMM [15].

An eight-camera Vicon MX Motion Capture System (Vicon Motion Systems Ltd., Oxford, UK) was used to capture the position of 17 reflective markers at 100 Hz. We used specialized software (Vicon Nexus 1.8.5, Vicon Motion Systems Ltd., Oxford, UK) to build anthropometric model of the legs and feet of the subject and visualize the three-dimensional position of the markers in the global coordinate system of the gait-analysis laboratory. The raw position data for each marker were exported as .csv files from Nexus for statistical analysis.

### 2.3. Data Analysis

Each subject was required to take more than ten steps over 10 meters. Incomplete gait cycles at the initiation and termination of each trial were excluded, and the remaining gait cycles were analyzed. We normalized each gait cycle to 100 timepoints by linear interpolation to make data comparable among subjects.

#### 2.3.1. Preprocessing

Preprocessing and spatiotemporal gait characteristics were conducted using a custom program written in MATLAB R2018a (MathWorks, Inc., Massachusetts, USA). Specifically, the motion data were filtered by a low-pass, zero-phase-shift, first-order *Butterworth* filter with no more than 1 dB of ripple in the passband from 0 to 0.01 Hz and at least 3 dB of attenuation in the stopband above 20 Hz.

#### 2.3.2. Gait Cycle, Phases, and Rockers

A complete gait cycle included the *stance phase* and *swing phase*. When the heel struck the floor, the dorsal calcaneus (CCL) reached the minimal *z*-axis value. This moment was the beginning of a new gait cycle; the toe was then lowered gradually to the floor, gripping forcefully until toe-off during the stance phase. We used the *z*-axis minimal value of the hallux (HLX) marker in the gait cycle to divide the stance and swing phases.

The stance phase was further divided into three *rocker phases*: the first rocker phase was from heel-strike to foot-flat; the second rocker phase was from foot flat to heel-off; and the third rocker phase was from heel-off to toe-off. The gait cycles, phases, and rockers were split according to the method described below and shown in Figure 2.

The first rocker phase was from heel-strike to foot-flat. During this phase, plantar flexion increased until the distal end of the metatarsal (DMT) marker reached the floor. The second rocker phase was from foot-flat to heel-off. During this phase, the foot lay flat on the floor, and the CCL maintained a stable position in the *z*-axis (with an interframe difference < 1 mm) except for a few minor tremors caused by elastic deformation of the skin during dorsiflexion. When the third rocker phase began (the heel-off), the interframe difference increased rapidly (interframe difference ≥ 1 mm), and the CCL position in the *z*-axis increased quickly in the third rocker phase until toe-off.

#### 2.3.3. Basic Gait Parameters

Stride length measured the distance between the CCL points of two consecutive footprints of the same side, and the stride duration referred to the elapsed time between first heel strikes of two consecutive footfalls of the same side. The first/second/third rocker percentages were the elapsed time percentages of the first/second/third rocker phases in the gait cycle in this work. The stance/swing phase percentage was the elapsed time percentage of the stance/swing phase in the gait cycle.

#### 2.3.4. Velocity Profiles

The velocity of any given marker was calculated by examining the change in displacement over time on the line of progression. Five markers were chosen for calculating velocity profiles at different joints, including the tibial tuberosity (TTU, knee), lateral malleolus (LML, ankle), CCL (back foot), the distal end of the second metatarsal (DMT2, front foot), and the HLX (tip of foot). These markers were largely independent of each other and were considered clinically relevant as they can reveal pathologic features of the gait after LCL injuries to the ankle [15].

For each marker, we reported the maximal velocity (*V*_max_) in the gait cycle, the minimal velocity (*V*_min_) in the gait cycle, the time from the start of the gait cycle to maximal velocity (TV_max_), and the time from the start of the gait cycle to minimal velocity (TV_min_).

#### 2.3.5. Acceleration Profiles and Microadjustments

Different joints in the legs and feet of the subject moved with different speeds over different phases of a gait cycle. The definitions of acceleration and microadjustment are displayed in Figure 3. Changes in velocity (speeding up or slowing down) can be described by acceleration. The microadjustment is derived from acceleration. Acceleration was defined as the rate of change in velocity over time. In an acceleration curve, the acceleration dropped to zero was counted as a *microadjustment*. The microadjustment from acceleration to deceleration was defined as a *peak* in the velocity, and the microadjustment from deceleration to acceleration was defined as a *valley* in the velocity. Microadjustments reflected the postural control in the lower limb.

#### 2.3.6. Statistical Analysis

The Shapiro-Wilk's test (*p* > 0.05), a visual inspection of histograms, and normal Q-Q plots (Quantile-Quantile Plots) showed that spatiotemporal gait variables—including temporal variables, velocities, and microadjustments—were approximately normally distributed.

A one-way analysis of variance (ANOVA) was conducted to compare gait cycles between ligament-injury patients and control subjects. The number of microadjustments were then compared among five markers using a one-way repeated ANOVA and least significance difference (LSD) post hoc multiple-comparison test to examine differences over different leg and foot joints.

We performed statistical analyses using SPSS, v. 25.0 (IBM Corp., Chicago, USA). The mean and standard error (SE) with an a priori level of 0.05 are reported in this paper.

## 3. Results

A total of 30 injury-gait cycles were successfully collected from three patients diagnosed with LCL injuries of the ankle before surgery (all male, with a mean age of 34 years [range, 32–37]; BMI, 26.39 ± 4.64 [mean ± SD]). The average time since the last sprain in the injury group was 19 weeks. All patients were treated and recommended by one surgeon specializing in sports medicine. Fifty normal-gait cycles were also collected from three control subjects (all male, mean age 26 years [25–28]; BMI, 19.07 ± 3.46). In the control subjects, gait recorded from both legs was mixed and compared to gait recorded from the affected side in the LCL-injury patients.

### 3.1. Gait Analysis

On average, ligament-injury patients walked slower and took smaller strides than control subjects. Specifically, stride length was reduced from 1419.8 mm to 1330.7 mm (*p* < 0.001), and stride duration was increased from 0.98 to 1.08 s/stride (*p* < 0.001, Table 1).

### 3.2. Phase Differences

Patients exhibited a significantly shorter percentage in the first rocker phase (4.67% vs. 6.76%, *p* < 0.001) and longer in the second rocker phase (25.80% ± 0.39 vs. 24.26% ± 0.38, *p* = 0.009; Table 1) than the control subjects. We did not find significant differences in the third rocker phase (*p* = 0.656), neither in stance phases nor in swing phases (*p* = 0.849).

### 3.3. Velocity Profiles

Leg velocity profiles are displayed in Table 2 and Figure 4. As shown in Table 2, *V*_max_ recorded from five selected markers was significantly different between the two groups; patients' maximal velocity was higher than that of the control subjects (Figure 4). TV_max_ recorded from LML, CCL, DMT2, and HLX displayed significant differences between patients and control subjects; specifically, patients reached peak velocity later than the control subjects. The *V*_min_ recorded from TTU, LML, and DMT2 displayed a significant difference between patients and control subjects; in these markers, *V*_min_ was higher in patients than in the control subjects. TV_min_ only showed significance in data collected at TTU, where control subjects reached a minimal velocity later than patients.

### 3.4. Acceleration Profiles and Microadjustments

To quantify the efforts in maintaining stability, we measured the number of microadjustments performed by patients and control subjects during the three rockers and the swing phase (Table 3). Compared to control subjects, patients with ligament injuries produced more microadjustments in the stance phase but not the swing phase. The only significant difference occurred in the second rocker phase (4.87 ± 0.54 vs. 3.20 ± 0.38, *p* = 0.017). In this phase, the knee, ankle, and metatarsal of patients exhibited a significant more valleys in velocity; the knee, ankle, calcaneus, and metatarsal of patients exhibited a significant more peaks in velocity; and the knee, ankle, calcaneus, metatarsal, and hallux of patients showed a higher mean velocity (Table 4).

In addition to the comparison between patients and control subjects, we investigated differences among five different joints. As displayed in Table 5, subjects displayed different microadjustment behaviors among five joints, and such differences among joints were altered at the walk phases of stance and swing.

Specifically, in the first rocker phase, the knee (1.08), ankle (1.00), and calcaneus (1.00) displayed more microadjustments than the metatarsal (0.33) and hallux (0.17). In the second rocker phase, a significantly larger number of microadjustments occurred in the metatarsal (6.33), ankle (4.83), and calcaneus (3.83) than in the hallux (3.00) and knee (2.17). In the third rocker phase, a significantly larger number of microadjustments occurred in the metatarsal (3.50) and hallux (5.17) compared to the knee (0.17), ankle (0.17), or calcaneus (0.17). In the swing phase, a significantly larger number of microadjustments occurred in the knee (2.50) and calcaneus (2.50) compared to the metatarsal (1.50), hallux (1.67), and ankle (1.00).

## 4. Discussion

A three-dimensional motion-tracking system was used to investigate whether LCL-injury patients displayed certain types of gait patterns with unique spatiotemporal characteristics during gait cycles. Our research hypothesis patients with ligament injury would exhibit a shorter stance phase that was supported by our experimental results (Table 1). Patients with LCL injuries of the ankle exhibited a shorter stance phase due to the pain surrounding their ankle when their feet touched the ground. They decreased stride length and increased stride duration compared to control subjects. Upon further examination, we noted significant differences in the gait cycle during the first and second rockers, wherein patients exhibited a briefer time to move their body mass from the hindfoot to the forefoot (Table 1, Figure 2).

Other researchers also reported this phenomenon. Khazzam et al. reported that compared with normal subjects, patients with degenerative diseases of the foot revealed a shortened stride length, reduced cadence, and decreased walking speed [16]. Patients with chronic ankle instability also displayed lower gait velocity, lower cadence, and smaller step length [17]. Meng et al. demonstrated that the sound limb of patients with LCL injuries of the ankle compensated for the affected side, to reduce the load on the affected side by switching quickly to the phase of vertical support at the moment of heel strike [18]. Ligament injuries surrounding the ankle may thus be the root cause of the quick shift in weight-bearing.

Our research hypothesis patients with ligament injury would manifest a relatively slower velocity were also supported. Patients increased maximal and minimal velocities in their knee, ankle, and foot during the gait cycle. Evidence from Table 2 and Figure 4 indicated that a larger deviation in velocity profiles of patients occurred during the second rocker phase compared to the control subjects. This observation aligned with the increasing difficulty in maintaining the stability of the foot and ankle after injuries to the surrounding ligaments.

By examining the acceleration profiles, we found that LCL-injury patients performed more microadjustments than the control subjects, especially in the second rocker phase. When the calcaneus touches the floor during the early stance phase, the musculoskeletal structure of the foot and ankle accepts force immediately; ligaments surrounding the ankle then need to work in coordination to provide stable support. In the case of LCL injuries to the ankle, such coordination may be partially disturbed, which may cause the microadjustments that we observed in patients during the early stance phase (Tables 3 and 4). As body weight moves forward, the epicenter of microadjustments shifts from the proximal to distal limb and from the back to the front foot (Table 5).

The increasing number of microadjustments observed in the stance phase of the LCL-injury patients was a novel finding in this study. Previous investigators found that individuals with chronic ankle instability displayed balance deficits as measured by kinematic balance analysis [19, 20]. Konradsen et al. suggested that the feedforward mechanism or activation was crucial in preparing joint loading as muscle preactivation influenced joint stiffness [21]. Feedback loops also play an equally important role in making rapid adjustments during walking, and any deficit in the feedforward and/or feedback mechanism leads to impaired neuromuscular control [22–25]. Proprioception loss in patients with ankle instability also disturbs their instant detection of joint position [26, 27]. The impaired neuromuscular control resulting from LCL injuries of the ankle then places the patients at risk of sustaining an ankle sprain, and a maladaptive position of the foot before touching down on the floor can lead to ankle re-injury [28, 29].

Combining evidence from other previous studies and our findings, we provide a more comprehensive explanation as to why some patients frequently twist their ankles again after their first injury. A deficiency in feedforward and feedback loops of LCL-injury patients leads to increasing numbers of microadjustments of the foot during the early stance phase in walking, and when interference occurs due to uneven terrain or an unexpected perturbation, ankle twists may occur repeatedly [30].

Another intriguing finding of the current study was the different velocity profiles of patients during the early swing phase. As shown in Figure 4, patients displayed lower velocities than control subjects, especially from the forefoot (Figure 4, fourth and fifth rows), while the knee velocity profiles of the patients were similar to the control subjects during the swing phase (Figure 4, first row). These results suggest that there is some underlying protective mechanism at work in the early swing phase that reduces the velocity of the subtalar joint of the LCL-injured patients.

### 4.1. Implications

Knowledge learned from the microadjustments analyzed in this study can help us to design protective measures for LCL-injury patients during the early stance phase, such as designing a special cushion to release force and loads after the calcaneus touches the floor. We can also use microadjustments as a measure to evaluate the outcome of surgical intervention.

A detailed description of spatiotemporal gait characteristics will also improve our future attempts at identifying a pattern of ligament injury by using artificial-intelligence technologies [31–33]. For example, multisegmental, three-dimensional motion data collected by the HFMM can be analyzed by machine learning/deep-learning algorithms. We expect that in the future, specific spatiotemporal- and kinematic feature-based HFMM will support intelligent assessment of locomotor function based upon patient gait differences and thus provide treatment consultation for patients with ligament injuries.

### 4.2. Limitations

Several limitations of the current analysis need to be addressed, the first of which came from our participants. Patients and control subjects consisted of young males only. Thus, the sample size needs to be increased in the future and should include female patients and control subjects. The second limitation was that participants were only asked to walk on a flat surface without adding a stairway, as most other gait studies have done [34, 35]. These two factors limit the generalizability of our findings, and caution must thus be exercised when applying our results to other gait-study settings.

## 5. Conclusions

Our findings revealed that patients with LCL injuries of the ankle displayed a shorter stride length, slower stride in the gait cycle, and more microadjustments than control subjects. The above observations are more significant in the second rocker phase than in other rocker/swing phases. Evidence from velocity profiles suggested that patients with ligament injury necessitated more musculoskeletal microadjustments to maintain body balance, but these adjustments may also be due to secondary injury. Precise descriptions of the spatiotemporal gait characteristics are therefore crucial to our understanding of movement control during locomotion and can also serve as an assessment tool for surgical and rehabilitative management.

## Figures and Tables

**Figure 1:** (a) Tracking movements of subjects using a Vicon MX Motion Capture System. (b) Marker placement based on HFMM. LEP/MEP, lateral/medial epicondyle; TTU: tibial tuberosity; SH1/2: two points on the medial side of the tibia; LML/MML: lateral/medial malleolus; LCL/CCL/MCL: lateral/dorsal/medial calcaneus; NAV: navicular; PMT1/PMT5: proximal end of the first and fifth metatarsals; DMT1/2/5: distal end of the first/second/fifth metatarsals; HLX: hallux.

**Figure 2:** Gait cycles, phases, and rocker splitting.

**Figure 3:** Velocity, acceleration, and microadjustments of LML in a gait cycle.

**Figure 4:** Velocity profiles of five anatomic landmarks (in rows, marked by five sensors: TTU, LML, CCL, DMT2, and HLX) over the entire gait cycles of three patients (in columns). Please note that each gait cycle was normalized to time, and three long vertical lines separate the phases. On each marker, the mean velocity profile (solid lines) over ten strides of the patient is displayed above the 50 velocity curves (gray dots) taken from three normal participants.

**Table 1:** Basic measures to the gait cycle.

Basic parameter	Patients (*n* = 30, gait cycle #)	Controls (*n* = 50, gait cycle #)	*p* value
	Mean ± SE	Mean ± SE	
1^st^ rocker percentage (%)	4.67 ± 0.15	6.76 ± 0.16	**<0.001**
2^nd^ rocker percentage (%)	25.80 ± 0.39	24.26 ± 0.38	**0.009**
3^rd^ rocker percentage (%)	28.50 ± 0.88	28.12 ± 0.40	0.656
Stance phase percentage (%)	58.97 ± 0.88	59.14 ± 0.20	0.849
Swing phase percentage (%)	41.03 ± 0.88	40.86 ± 0.20	0.849
Stride length (mm)	1330.7 ± 6.35	1419.8 ± 7.46	**<0.001**
Duration (s/stride)	1.08 ± 0.01	0.98 ± 0.01	**<0.001**

**Table 2:** Velocity measurements in the gait cycle.

Marker	Parameter in GC	Patients (*n* = 30, gait cycle #)	Controls (*n* = 50, gait cycle #)	*p* value
		Mean ± SE	Mean ± SE	
TTU	*V*_max_ (mm/10^−2^s)	30.73 ± 0.43	27.95 ± 0.20	**<0.001**
	TV_max_ (%)	66.57 ± 0.40	66.62 ± 0.39	0.929
	*V*_min_ (mm/10^−2^s)	3.48 ± 0.21	1.77 ± 0.05	**<0.001**
	TV_min_ (%)	22.07 ± 0.76	24.28 ± 0.23	**0.009**

LML	*V*_max_ (mm/10^−2^s)	45.06 ± 0.57	42.35 ± 0.30	**<0.001**
	TV_max_ (%)	85.33 ± 0.23	82.92 ± 0.24	**<0.001**
	*V*_min_ (mm/10^−2^s)	0.26 ± 0.02	0.12 ± 0.01	**<0.001**
	TV_min_ (%)	16.50 ± 0.70	16.74 ± 0.60	0.801

CCL	*V*_max_ (mm/10^−2^s)	47.15 ± 0.74	43.59 ± 0.29	**<0.001**
	TV_max_ (%)	84.80 ± 0.22	83.06 ± 0.19	**<0.001**
	*V*_min_ (mm/10^−2^s)	0.14 ± 0.01	0.12 ± 0.01	0.134
	TV_min_ (%)	13.83 ± 0.56	12.54 ± 0.47	0.087

DMT2	*V*_max_ (mm/10^−2^s)	47.76 ± 0.68	44.41 ± 0.27	**<0.001**
	TV_max_ (%)	83.77 ± 0.33	81.66 ± 0.21	**<0.001**
	*V*_min_ (mm/10^−2^s)	0.13 ± 0.01	0.09 ± 0.01	**0.002**
	TV_min_ (%)	29.50 ± 2.04	28.40 ± 1.27	0.650

HLX	*V*_max_ (mm/10^−2^s)	49.03 ± 0.77	44.95 ± 0.26	**<0.001**
	TV_max_ (%)	82.50 ± 0.43	79.44 ± 0.42	**<0.001**
	*V*_min_ (mm/10^−2^s)	0.07 ± 0.01	0.08 ± 0.00	0.600
	TV_min_ (%)	42.83 ± 1.86	39.78 ± 1.91	0.255

Notes: TTU: tibial tuberosity; LML: lateral malleolus; CCL: dorsal calcaneus; DMT2: distal 2^nd^ metatarsal; HLX: hallux; *V*_max_: maximal velocity; *V*_min_: minimal velocity; TV_max_: time to maximal velocity; TV_min_: time to minimal velocity.

**Table 3:** Microadjustments to the gait cycle.

No. of microadjustments	Patients (*n* = 30, gait cycle #)	Controls (*n* = 50, gait cycle #)	*p* value
	Mean ± SE	Mean ± SE	
1^st^ rocker (#)	0.87 ± 0.14	0.57 ± 0.10	0.097
2^nd^ rocker (#)	4.87 ± 0.54	3.20 ± 0.38	**0.017**
3^rd^ rocker (#)	2.00 ± 0.24	1.67 ± 0.17	0.273
Swing phase (#)	1.80 ± 0.14	1.87 ± 0.10	0.696

**Table 4:** Velocity measurements in the 2^nd^ rocker phase.

Marker	Parameter in 2^nd^ rocker	Patient (*n* = 30, gait cycle #)	Control (*n* = 50, gait cycle #)	*p* value
		Mean ± SE	Mean ± SE	
TTU	No. of valleys (#)	2.47 ± 0.23	1.16 ± 0.07	**<0.001**
	No. of peaks (#)	1.87 ± 0.25	0.22 ± 0.06	**<0.001**
	Velocity (mm/10^−2^s)	6.05 ± 0.07	4.74 ± 0.08	**<0.001**

LML	No. of valleys (#)	3.73 ± 0.19	3.16 ± 0.12	**0.007**
	No. of peaks (#)	2.97 ± 0.17	2.34 ± 0.13	**0.004**
	Velocity (mm/10^−2^s)	0.85 ± 0.03	0.52 ± 0.02	**<0.001**

CCL	No. of valleys (#)	3.37 ± 0.19	2.94 ± 0.17	0.106
	No. of peaks (#)	2.67 ± 0.18	2.14 ± 0.16	**0.040**
	Velocity (mm/10^−2^s)	0.54 ± 0.02	0.57 ± 0.03	0.404

DMT2	No. of valleys (#)	3.80 ± 0.34	3.02 ± 0.13	**0.041**
	No. of peaks (#)	3.50 ± 0.35	2.36 ± 0.13	**0.005**
	Velocity (mm/10^−2^s)	0.79 ± 0.03	0.48 ± 0.01	**<0.001**

HLX	No. of valleys (#)	2.10 ± 0.17	2.28 ± 0.12	0.372
	No. of peaks (#)	1.67 ± 0.17	1.60 ± 0.12	0.740
	Velocity (mm/10^−2^s)	1.72 ± 0.10	0.97 ± 0.04	**<0.001**

Notes: TTU: tibial tuberosity; LML: lateral malleolus; CCL: dorsal calcaneus; DMT2: distal 2^nd^ metatarsal; HLX: hallux.

**Table 5:** Number of segmental microadjustments during the three rockers and swing phase.

No. of microadjustments	TTU	LML	CCL	DMT2	HLX	SE	*p* value
	Mean	Mean	Mean	Mean	Mean		
1^st^ rocker (#)	1.08	1.00	1.00	0.33	0.17	0.20	**0.003**
2^nd^ rocker (#)	2.17	4.83	3.83	6.33	3.00	0.74	**0.004**
3^rd^ rocker (#)	0.17	0.17	0.17	3.50	5.17	0.34	**< 0.001**
Swing phase (#)	2.50	1.00	2.50	1.50	1.67	0.19	**< 0.001**

Notes: TTU: tibial tuberosity; LML: lateral malleolus; CCL: dorsal calcaneus; DMT2: distal 2^nd^ metatarsal; HLX: hallux.

## Data Availability

This study was conducted at the motion analysis laboratory of the Peking University Third Hospital. The data in our study are not freely available because of patient privacy.
